# A Literature Review Research on Monitoring Conditions of Mechanical Equipment Based on Edge Computing

**DOI:** 10.1155/2022/9489306

**Published:** 2022-10-08

**Authors:** Liqiang Song, Huaiguang Wang, Zhiyong Shi

**Affiliations:** Department of Vehicle and Electrical Engineering, Shijiazhuang Campus, Army Engineering University of PLA, Shijiazhuang 050003, China

## Abstract

The motivation of this research is to review all methods used in data compression of collected data in monitoring the condition of equipment based on the framework of edge computing. Since a large amount of signal data is collected when monitoring conditions of mechanical equipment, namely, signals of running machines are continuously transmitted to be crunched, compressed data should be handled effectively. However, this process occupies resources since data transmission requires the allocation of a large capacity. To resolve this problem, this article examines the monitoring conditions of equipment based on edge computing. First, the signal is pre-processed by edge computing, so that the fault characteristics can be identified quickly. Second, signals with difficult-to-identify fault characteristics need to be compressed to save transmission resources. Then, different types of signal data collected in mechanical equipment conditions are compressed by various compression methods and uploaded to the cloud. Finally, the cloud platform, which has powerful processing capability, is processed to improve the volume of the data transmission. By examining and analyzing the monitoring conditions and signal compression methods of mechanical equipment, the future development trend is elaborated to provide references and ideas for the contemporary research of data monitoring and data compression algorithms. Consequently, the manuscript presents different compression methods in detail and clarifies the data compression methods used for the signal compression of equipment based on edge computing.

## 1. Introduction

Mechanical equipment was monitored to detect whether a mechanical failure occurred or not in the previous investigations, which is fairly a simple method to deal with monitoring mechanical failures. However, before a failure occurred, the machinery could have signaled to have stepped into serious failure mode. To resolve this issue, the first implemented attempt was the signal processing technology [1] that was developed and applied to the process of mechanical fault diagnosis [2]. However, the amount of signal data collected was increasingly large. To reduce the energy loss in data transmission and the size of data transmitted, data compression technology has been effectively applied in monitoring processes [3].

Data compression is a generic name that encodes data to squeeze [4], mainly representing high-frequency characteristics with shorter codes, like Shannon–Fano coding [5] and Huffman coding [6]. Data compression is divided into two compression methods, which are called lossless and lossy compressions, respectively, according to the quality of compression. The lossless compression is used when the reconstructed signal is required to be consistent with the original signal, such as arithmetic coding [7], dictionary coding [8], and run-length encoding (RLE) [9], is usually employed for text and some signal data with high fidelity. When the reconstructed signal needs a higher compression ratio (CR) under the premise of meeting the demand, lossy compression can be utilized, such as the threshold denoising processing method [10], compression methods based on data transformation [11], and mostly for signal data related to vibration analysis and sensing signals.

Even though data can be compressed well through compression methods, powerful computing ability is required in this process when an increase in the complexity of algorithms is encountered. So, hardware becomes the key component to improve the capability of the algorithm. The development of data processing technology based on edge computing [12, 13] makes it possible to improve computing power. Therefore, edge computing is used for the transfer of user-side data, applications, and some services from the cloud to the edge of the network [14], which provides a more feasible solution for the data pre-processing task in state monitoring. By pre-processing the data right at the source where it is generated, it is possible to process signals quickly on the one hand and reduce the amount of data transmission, on the other hand, ensuring the low bandwidth and energy consumption required for transmission. Since the edge nodes already have some pre-processing capabilities, the burden of data processing on the cloud is greatly reduced, making the monitoring process timelier and more accurate.

To monitor the signal condition of mechanical equipment, the first step is to classify the status signal, which currently contains signals changing slowly and changing rapidly [15]. While a slowly changing signal refers to the measured signal data with a certain degree of continuity, or even a longer period to maintain the same status, the rapidly varying signal is a time-varying non-smooth signal with the characteristics of sudden change and discontinuity. Different data compression methods are chosen according to the types of monitored state signals. While lossless compression methods are used for slowly varying signals, lossy compression methods are employed for rapidly varying signals.

The rest of the article is organized as follows: Section 2 introduces the investigation of data pre-processing based on edge computing, then the available compression methods according to the monitoring condition characteristics of signals employing different mechanical equipment are introduced. The assessment indexes used by various compression methods in data compression methods are presented in Section 3. Section 4 discusses the future directions of these methods. Section 5 concludes the review research.

## 2. Monitoring Conditions Based on Edge Computing

### 2.1. Preliminary

Monitoring the status of equipment based on edge computing first contains the acquisition of signals, including slowly changing signals, such as water temperature and oil temperature, as well as fast-changing signals, such as engine vibration signals and transmission vibration signals. Then, the collected signals, and data, are pre-processed by edge computing, and the signals of the fault characteristics not easily identified are compressed and transmitted to the cloud for signal reconstruction and fault diagnosis. The whole signal analysis process is shown in Figure 1.

### 2.2. Pre-Processing of Data in Edge Computing

To avoid occupying a large number of transmission resources and energy loss, it is necessary to pre-process the data. In this article, we apply a pre-processing method based on edge computing to monitor the signal process of equipment status and extract the information of fault features through a short-time Fourier transform or wavelet transform [16], such as time domain characteristics of faults, frequency domain characteristics of faults and fault characteristics of the time–frequency domain, so that the fault information can be diagnosed quickly. However, not all fault information can be obtained by this method, such as identification based on high and low resonance components [17] and weak transient signal processing [18].

When signal data needs complex calculation, such as pulse signal, decay signal, noise signal, and other combined signal components, the data is transmitted to the cloud for analysis and calculation, therefore, we need to compress and transmit them, and decompose the signal and identify the fault characteristics in the cloud for such data types.

## 3. Data Compression Methods for Collected Mechanical Signals

Different processing methods are required for compression based on the signal type. If the sampling frequency of fast-varying signals is too high, the amount of data collected will be very large, resulting in a large amount of transmitted data. A lossless compression algorithm can compress them, but it cannot meet the CR required for the fast-varying signal, so lossy compression is applied to the fast-varying signal compression since a lossless compression algorithm is used for slow-varying signals.

### 3.1. Lossless Compression Method for Slowly Varying Signals

Due to the small variability occurring in slow-varying signals over a short period, the amplitude of the remaining numbers is significantly reduced by the differential transformation of the data, which results in a lower number of binary bits required for representation. This implies that lossless compression is more effective. Lossless compression was initially used in data monitoring algorithms based on a single compression algorithm, which is more effective regarding the computational complexity, but its CR is less than expected. To improve its compression effect, multiple compression algorithms need to be utilized in combination, so numerous hybrid algorithm compression models have been suggested, which have the advantage of improving further the CR of the data. However, the complexity of the algorithm increases.

#### 3.1.1. Single-Algorithm Data Compression Model

The single-algorithm model mainly includes statistical-based and dictionary-based compression algorithms. While statistical-based compression algorithms compress data by counting the frequency of characters and providing fewer bits of encoding for characters with high frequency, the dictionary-based compression algorithm compresses data by constructing a dictionary and outputting its dictionary index value, which can be adapted to various types of data.

#### 3.1.2. Data Compression Model of the Hybrid Algorithm

When the hybrid algorithm compression models are under consideration, one type is based on the improved compression algorithm, such as moving to front (MTF) coding [19], Burrows–Wheeler Transform (BWT) coding [20], and XOR incremental coding [21] to realize a better sequence that is more suitable for compression, to improve CR with the combination of single-algorithm code.

The other type is a compression method that combines different single-algorithm models, mainly through a mixture of statistical-based compression algorithms and dictionary-based compression algorithms, which outputs its index value through the dictionary coding and compress data through a statistical-based encoding algorithm.  Table 1 presents different algorithms and their advantages and disadvantages of each.

Through the analysis of the various lossless compression methods in Table 1, the mixed compression algorithm can be used to compress slowly changing signals collected by monitoring equipment, and the LZW algorithm can finitely compress the data while outputting its encoding, and then the finite state entropy compression algorithm can obtain a better compression effect. On the other hand, how to improve the shortcomings of the LZW algorithm to enhance compression efficiency will be a key research direction for researchers.

### 3.2. Lossy Compression Method for Rapidly Varying Signals

When monitoring equipment is conducted, the most applied mechanical vibration signal is analyzed to understand the operation status of the equipment. In this article, vibration signal analysis is employed as an example to investigate and review the compression algorithms. After the vibration signal is collected, the fault signal is detected by edge computing to extract more effective signal information. Then, the research on the lossy compression algorithm is carried out on this basis. At present, there have been many studies dealing with lossy compression algorithms for vibration signals, but they have not been classified yet.

In this research, lossy compression methods for vibration signals are studied and classified to present their research directions. In the early stage, the quantization compression algorithm has higher efficiency, but the CR is not high. To improve its compression effect, one method applied is based on decomposing signals to extract its effective components and remove invalid components. Therefore, the removal methods include threshold processing and correlation analysis, such as empirical mode decomposition (EMD) [33] and improved algorithms ensemble empirical mode decomposition [34, 35] complete ensemble empirical mode decomposition with adaptive noise [36, 37], intrinsic time-scale decomposition (ITD) [38, 39], and local mean decomposition [40]. The other type is the sparse transformation of signals, which is conducted by constructing complete dictionaries and super-complete dictionaries [41]. Although the complete dictionary can reduce the sparsity of the signal to a certain extent, it is difficult to achieve the complete decomposition of the signal by a single dictionary for different components contained in the original signal, such as shock signal and simple harmonic signal.

Therefore, the super-complete dictionary is studied [42], which is employed for the sparse decomposition of signals. How to realize the orthogonalization of atoms in the construction of the super-complete dictionary and how to establish a more excellent sparsification method are still open research directions to investigate.

With the development of deep learning technology, compression algorithms based on deep learning have also been studied in more detail, such as recurrent neural network-based recurrent neural networks (RNN) [43] and long short-term memory algorithm [44, 45]. By mapping the original signal to the implicit layer as well as the pooling layer, pruning techniques are researched [46]. The effective components of the signal are preserved, which makes the data transmission reduced.

Although the single-algorithm compression model can effectively reduce the redundancy of data and improve the CR, there exists still room for the improvement of the CR. By studying the compression model based on a hybrid algorithm utilizing the single algorithm, the signal is first decomposed or sparsely transformed and then compressed using lossless compression methods. So, its algorithm can further improve the CR, but its computational complexity increases. Lossy compression methods and their advantages and disadvantages are described in Table 2.

By comparing the advantages and disadvantages of the data compression methods in Table 2, the compression method based on sparse transform can decompose the fast-varying signal sparsely, and a more effective sparse signal can be obtained through a dictionary employing orthogonal transformation to improve the CR, and then the algorithm of finite state entropy is utilized to further process data to obtain a better-compressed signal.

## 4. Evaluation Metrics Used by Data Compression Methods

The performance of the data compression algorithm needs to be evaluated by establishing a corresponding evaluation index. The number of the current compression algorithm evaluations related to the lossless method is relatively few, which is mainly due to the original signal and reconstruction signals remaining the same, so there occurs no data loss. Therefore, the lossless compression algorithm is mainly evaluated through the CR and time. The greater the CR is, the more effective the compression would be, the shorter the compression time is, the lower the complexity of the algorithm would be, and the better the processing of data would be. The formula for its CR is defined by

(1) $$\begin{array}{c} \text{CR}=\frac{{\text{Data}}_{0}}{{\text{Data}}_{1}}, \end{array}$$

where Data_0_ denotes the bit number of original data and Data_1_ denotes the bit number of compressed data.

Since lossless compression needs to ensure the consistency between the original data and the reconstructed data, it limits the increase of the CR, and many optimization algorithms have still been struggling to improve the performance of the CR.

Unlike lossless compression, the reconstructed signal in lossy compression methods does not need to be consistent with the original signal, so in addition to the CR and time, the fidelity of its signal needs to be evaluated. The corresponding evaluation indexes are presented as follows [63].

### 4.1. Root Mean Square Error (RMSE)

The RMSE method quantifies the degree of data distortion caused by the compression algorithm. When the RMSE value nears zero, the original signal is consistent with the reconstructed signal and there is no compression effect.

(2) $$\begin{array}{c} \text{RMSE}=\sqrt{\frac{1}{N}\overset{N}{\underset{i=1}{\sum }}{\left(x_{i}-x_{i}^{r}\right)}^{2}}\times 100, \end{array}$$

where *x*_*i*_ and *x*_*i*_^*r*^ are the original signal and the reconstructed signal, respectively and *N* is the amount of signal data.

### 4.2. Percent Root Mean Square Difference (PRD)

To reduce the influence of the signal mean on the RMSE, a normalized PRD is established, thus disregarding the influence of its mean, which is given by

(3) $$\begin{array}{c} \text{PRD}=\sqrt{\frac{\overset{N}{\underset{i=1}{\sum }}{\left(x_{i}-x_{i}^{r}\right)}^{2}}{\overset{N}{\underset{i=1}{\sum }}{\left(x_{i}-\bar{x}\right)}^{2}}}\times 100. \end{array}$$

### 4.3. Signal-to-Noise Ratio (SNR)

It is used to evaluate the similarity between the original signal and the reconstructed signal by

(4) $$\begin{array}{c} \text{SNR}=10\times \log_{10}\left(\frac{\overset{N}{\underset{i=1}{\sum }}{\left(x_{i}-\bar{x}\right)}^{2}}{\overset{N}{\underset{i=1}{\sum }}{\left(x_{i}-x_{i}^{r}\right)}^{2}}\right). \end{array}$$

To understand whether there is a loss of key features when performing fault feature extraction before and after compression, it is necessary to compare the fault feature information before and after compression to ensure that useful fault features can be extracted from the reconstructed signal even though the evaluation metrics above for lossy compression are employed. The current study of fault features requires the examination of fault information in the time domain, frequency domain, and time–frequency domain [64]. Lei and Zuo [65] classified their faulty signals, and selected their key information for fault diagnosis so that the corresponding information could be identified in the reconstructed signal, and thus discern the fidelity of their compressed data by comparing the key information in the original signal with the reconstructed signal.

## 5. Future Directions

With the development of edge computing and data compression methods, monitoring mechanical equipment has become more practical and useful than ever. In this section, the progression trend of monitoring mechanical equipment and data compression algorithms will be presented in detail.

### 5.1. Development Trend of Monitoring Mechanical Equipment

With the development of automated equipment, the inspection of offline mechanical equipment using automated equipment was realized. However, this method has still a certain deficiency in the inspection process. Due to the development of signal processing technology and the emergence of intelligent technology, online remote monitoring of mechanical equipment in real time has become more possible and reliable. However, data collected in this process is all uplinked to the cloud for crunching. Although this processing satisfies the functional requirements to a certain extent, there has still been a certain delay.

The edge node is utilized by transferring the data processing from the cloud to the edge node, thus speeding up its downlink computational process. Moreover, the real-time capability of data monitoring is effectively improved by filtering out data, processing it, and uploading it to the cloud for analysis. So, the amount of signal data that needs to be compressed is effectively reduced, and so does the amount of data transmission.

Based on the development trend of smart methods, monitoring of mechanical equipment also contribute to the improvement of the miniaturization of its equipment. So, the development of microelectronics technology, such as the application of digital signal processing and field programmable gate array-based devices, has effectively improved its micro-processing capability. On the other hand, the development of communication technologies, such as Internet of Things [66] and 5G [67, 68] transfer the information processing capability from the edge node to the cloud more efficiently in equipment monitoring.

### 5.2. Development Trend of Data Compression Technology

When equipment is monitored, the signal data is compressed with the help of different compression methods due to the different characteristics of the signal data.

To improve the CR, the CR of the single algorithm is enhanced on the one hand, and the complexity of the hybrid compression algorithm is reduced on the other hand by employing the characteristics of slowly varying data.

In the single algorithm, the traditional compression method is algorithmically optimized to improve its compression performance. The algorithm proposed by Huffman is improved based on the adaptive Huffman coding [69] and weighted adaptive Huffman coding [70]. Besides, the optimization algorithms, such as arithmetic coding based on context-based binary arithmetic coding [71] and RLE based on adaptive run-length coding [72] are employed. Duda [74] proposed a new lossless compression algorithm called asymmetric numeral systems (ANS) [73], whose computational speed is better than that of Huffman coding, and its compression performance is near to arithmetic coding, which is better to remedy the lack of algorithm complexity and CR [74]. Therefore, it can improve the algorithm complexity and CR.

Based on the ANS algorithm, a finite state entropy algorithm was developed. To further improve the compression and decompression speed, an optimization algorithm called *Z*-standard combined with LZ77 [75] was developed for lossless compression. Due to the emergence of deep learning techniques, the encoder–decoder algorithm can effectively save the compression time after the model is trained, and thus it is also applied to the field of data compressions called the deep learning model [77] based on multiple processing layers and deep learning algorithms to adapt to various data types proposed by Hinton and co-workers [76]. Although this algorithm can improve the compression performance, the training of the preliminary model requires a dataset and a long computational time, so it has certain limitations.

In the hybrid compression algorithm, to meet the impact of real-time transmission and reduce the time consumed by compression, it is necessary to reduce the complexity of the algorithm. Many of the current algorithms [78, 79] are improved mainly based on the CR, and the complexity of its compression needs to be examined to satisfy the real-time requirements.

On the other hand, fast-varying signals are researched regarding lossy compression methods. Since it allows a certain information loss in reconstructed signals, the CR is much higher when compared to a lossless one. When signal processing technology is under consideration, compression methods based on signal processing have become the mainstream research direction, such as compression methods run by sparse processing or threshold processing algorithms based on signal decomposition.

In the compression method of sparse processing, the energy distribution of the data is more concentrated by employing entropy transformation, and the low-energy data are removed, and then quantization is performed. Then, the quantized data are encoded [80, 34]. The CR can be maximized, but how to reduce the computational complexity in the real-time monitoring system still needs to be investigated. Due to the development of deep learning technology, the deep learning neural network is introduced into the compression algorithms [81]. Although the pruning-based algorithm can improve the CR, there has still been room for a better compression process, so a hybrid algorithm combining sparse transform and deep learning [82] has been researched.

## 6. Conclusion

The motivation of this research is to review all methods used in data compression of collected data in monitoring the condition of equipment based on the framework of edge computing. This article introduces a literature review of various data compression methods based on edge computing, which pre-processes the collected signal through edge computing to obtain easily identifiable fault signals and then performs data compression that is not generally easy to conduct. Two key indicators, algorithm complexity and CR are paid attention to when the literature is reviewed.

Concluded that when signal processing technology is under consideration, compression methods based on signal processing have become the mainstream research direction, such as compression methods run by sparse processing or threshold processing algorithms based on signal decomposition equipped with deep learning technology.

The manuscript presents different compression methods in detail and clarifies the data compression methods used for the signal compression of equipment. Then, comprehensive classification is presented based on various assessment methods to determine the fidelity of the compression methods.

The future development trend of monitoring equipment and data compression is comprehensively provided by presenting several research findings in the literature. Consequently, more detailed references and ideas for data compression of equipment are summarized for interested readers.

## Figures and Tables

**Figure 1:** Signal analysis process of equipment monitoring.

**Table 1:** Lossless compression methods.

Compression algorithm model	Compression algorithm type	Algorithm title	Advantages	Disadvantages
Single-algorithm compression model	Statistical-based compression algorithms	Huffman	Fast calculation speed. The greater the frequency difference, the better the compression effect.	The decoding process is slow and easily influenced by file size.
		Arithmetic coding	Good compression effect.	Complex calculation process.
		RLE	The algorithm is simple and has a good compression effect when there are more repetitive characters.	When there are few repetitive characters, the compression effect is poor or has the opposite effect.
		Asymmetric digital systems (ANS) [22]	The compression rate is close to arithmetic coding. Compression speed is close to Huffman coding.	rANS requires shift decomposition and tANS requires form construction.
		Finite state (FSE) [23]	ANS-based algorithm with high compression performance	Need to build a table of finite state entropy
	Dictionary-based compression algorithm	LZ77 [24], LZSS [25], and LZO [26]	High compression efficiency and very fast decompression speed of LZO	Poor compression when repeated characters are far apart
		LZ78 [27]	No need for a search buffer and memory	Need to create dictionaries and manage them. Complex to compile
		LZW [8]	A simple method with a good compression effect and the second field of LZ78 encoding removed	The dictionary update process causes a reduction in compression ratio (CR)
Hybrid algorithm compression model	Improved compression-based algorithm	MTF + single algorithm [28]	Ability to improve the alignment of its data, output its index of alignment, and create a high CR	Good for finite data only, not easy to handle when contains more data
		BWT + single algorithm [29]	BWT makes full use of its sequential arrangement and has a better compression effect	The algorithm process includes sorting, which takes up some memory and increases the time used for compression
		XOR incremental encoding + single algorithm [30]	Incremental encoding reduces the range of variation in the original data and reduces the number of binary bits represented	When the adjacent data vary very much, its compression becomes worse
	Hybrid compression of different single algorithms	RLE + Huffman [31]	With both data effects, it can get a higher CR and faster compression speed	However, it is limited by two compression methods on the dataset
		RLE + LZW [32]	Better data compression. No duplicate characters are encoded in the dictionary	Increased risk of error codes when coding

**Table 2:** Lossy compression methods.

Compression algorithm model	Compression algorithm type	Algorithm title	Advantages	Disadvantages
Single-algorithm compression model	Quantization-based compression algorithm	Scalar quantification [47]	Simple method and fast processing	Distorted data
		Vector quantization [48, 49]	Better than scalar quantification	Limited distortion
	Compression algorithm based on signal decomposition (threshold processing)	EMD [34]	Fast signal decomposition and fast compression	Easy to generate IMFs overlap, resulting in signal distortion
		Intrinsic time-scale decomposition [38]	Better computational speed than EMD, high time–frequency resolution, the good compression effect	Due to linear interpolation, it is easy to distort the intersection position
		VMD [50]	High decomposition accuracy, better decomposition of IMFs, accurate reduction of redundant information	With boundary effects, the parameters have a large impact on the results
		LMD [51]	Better preservation of transient change information in the original signal	Still has endpoint effects and does not have fast algorithms
	Compression algorithms based on sparse dictionary transformations (complete and overcomplete dictionaries)	STFT [52]	Capable of fast time and frequency conversion	Low resolution at high frequencies, resulting in signal loss during compression
		DCT [53]	Fast processing time and good sparse transformation effect	The transformation method does not work with all signals
		DWT [54] and LSWT [55]	With better time–frequency resolution, the LSWT algorithm does not consume memory	Excessive layer decomposition can result in wasted computational resources
		Best orthogonal basis [56]	Able to obtain near-optimal signal representation	Sparse is less effective when the signal cannot be represented by orthogonal components
		Orthogonal matching pursuit [57, 58]	Fast convergence to get a better sparse signal	The vertical projection of the processed signal is non-orthogonal and the number of iterations increases
		Generalized morphological component analysis [59, 60]	Capable of adapting to different input signal types, improving calculation speed and signal separation accuracy	The parameters of the calculation need to be set in advance, and the set values of the parameters directly affect the results of the processing
	Neural-network-based algorithm	RNN [43]	Very strong nonlinear mapping, high compression ratio (CR)	Requires training in the model and high computational resource requirements
Hybrid algorithm compression model	Lossy single algorithm + lossless compression single algorithm	Based on signal decomposition and Huffman [61]	Furthermore, increase in CR, no secondary data loss due to the introduction of lossless compression	This causes the complexity of the algorithm to increase and the data compression time to increase
		Based on sparse dictionary transform and RLE [62]		

## Data Availability

Data supporting this research article are available from the corresponding author or first author on reasonable request.
